The article "Optimizing the Catheter Care and Maintenance Strategy of Short-Term Catheterization among Hospitalized Patients in Microbiological Approach" was retracted in 2024. Reasons: signs of a paper mill; suspected computer-generated content; unreliable results or conclusions; concerns about the data.

# Optimizing the Catheter Care and Maintenance Strategy of Short-Term Catheterization among Hospitalized Patients in Microbiological Approach

**DOI:** 10.1155/2020/1971324

**Published:** 2020-11-28

**Authors:** Xiaoqiong Peng, Wei Qian, Jingming Zhuang, Jing Zhang, Zhengping Wang, Lijuan Shen, Qing Chang, Xuefeng Gu, Junfeng Shi, Jiangang Hou

**Affiliations:** ^1^Department of Urology, Huashan Hospital, Fudan University, Shanghai 200040, China; ^2^Department of Surgery, Huashan Hospital, Fudan University, Shanghai 200040, China; ^3^Clinical Trials Unit, Jiading District Central Hospital Affiliated Shanghai University of Medicine & Health Sciences, Shanghai 201800, China; ^4^Shanghai General Practice Medical Education and Research Center, Jiading District Central Hospital Affiliated Shanghai University of Medicine & Health Sciences, 201800, China; ^5^Shanghai Key Laboratory of Molecular Imaging, Shanghai University of Medicine & Health Sciences, Shanghai 201318, China; ^6^Research Department, Shanghai University of Medicine & Health Science Affiliated Zhoupu Hospital, Shanghai 201318, China

## Abstract

**Objective:**

To optimize the allocation of nursing resources, we investigate an alternative strategy for indwelling catheter cleaning.

**Methods:**

The present study involved a total of 117 male patients and 54 female patients, who were catheterized after urinary surgery from Aug 2018 to Feb 2019. The samples of indwelling catheter cleaning solutions were divided by two parts for microbiological culture and microbiome analysis.

**Results:**

No pathogenic bacteria were observed in the microbiological culture of the indwelling catheter cleaning samples from 24 h-uncleaned group and 48 h-uncleaned group. The microbiome analysis also showed no significant difference in bacterial diversity and quantity of the indwelling catheter cleaning solutions between the two groups.

**Conclusion:**

The indwelling catheter cleaning for male after urinary surgery can be prolonged to 48 h. The result of this study provided reliable basis for optimizing the allocation of clinical nursing resources.

## 1. Introduction

Indwelling catheterization is one of the most common clinical diagnosis and treatment techniques [1]. But the subsequent catheter-associated urinary tract infection (CAUTI) has troubled medical staff for a long time. According to previous studies and reports, urinary tract infections currently account for 40% of nosocomial infections [2], and about 80% of them are caused by indwelling catheterization [3]. The risk factors for CAUTI include the patient's own factors, the catheter duration time, the operation of catheter implantation, the meatal care, and the unreasonable clinical use of antibacterial drugs. Especially the duration of the catheter is the most important factor for the occurrence of CAUTI [4]. Many research reports on different populations have suggested that the short duration of catheterization is beneficial compared to the longer one [5–7]. According to reports, the risk of urethral bacterial infection each day in people undergoing catheterization is about 5%, reaching 100% within 4 weeks. The longer the catheter stays in place, the higher the risk of infection [8]. Guideline for Prevention of Catheter-Associated Urinary Tract Infections 2009 issued by the Healthcare Infection Control Practices Advisory Committee (HICPAC) suggested “Do not clean the periurethral area with antiseptics to prevent CAUTI while the catheter is in place. Routine hygiene (e.g., cleansing of the meatal surface during daily bathing or showering) is appropriate (Category IB)” and “Further research is needed on optimal cleaning and storage methods for catheters used for clean intermittent catheterization” [9]. In clinical practice, catheter care is usually performed twice a day after defecation (ensure the catheter is also cleaned) or when needed. However, Centers for Disease Control and Prevention Guidelines wrote “Insufficient evidence to recommend daily or twice-daily cleansing with soap and water or povidone-iodine solution” [10]. These existing vague materials caused us to think. The cleaning fluid of urinary catheters has been changed from the use of traditional disinfectants to normal saline [11]. It is inferred from this that the large number of daily urinary catheter care work increases the workload of care, is it also redundant? The duration of indwelling urinary catheter is greater than 3 days, and the incidence of CAUTI will be greater than 20% [12]. From the perspective of the practical significance of reducing the risk of infection and the economics of nursing, is it necessary to clean the patients with indwelling short-term catheters frequently within 72 hours after surgery? This needs to be confirmed based on a precise medical method and the concept of evidence-based medicine.

The article "Optimizing the Catheter Care and Maintenance Strategy of Short-Term Catheterization among Hospitalized Patients in Microbiological Approach" was retracted in 2024. Reasons: signs of a paper mill; suspected computer-generated content; unreliable results or conclusions; concerns about the data.

Based on the above speculations, we tested and analyzed the catheter wipe liquids of 117 male and 54 female patients with indwelling short-term catheterization after urinary system surgery. The microbes around the catheter of patients with short-term indwelling catheters of different lengths of indwelling and different cleansing frequencies were compared, which provided a specific biological basis for the improvement of indwelling catheter cleansing strategies.

## 2. Methods and Materials

### 2.1. General Information

We continuously collected data on patients with who were catheterized after urinary surgery from Aug 2018 to Feb 2019 in the Department of Urology, Huashan Hospital, Fudan University. Patients who did not meet all three of the following criteria were excluded: (1) indwelling catheter after surgery; (2) clear mind, normal communication; (3) agree to be involved in this study. The samples of precleaning and postcleaning were collected and classified according to the operation, the time of indwelling catheter, and the cleaning frequency (Table 1).

### 2.2. The Method of Indwelling Catheter Cleaning and Sampling

The method of indwelling catheter cleaning and sampling was standardized by using sterilized saline water to clean the surrounding area of urinary meatus, surface of catheter, and the area of 10 cm down to urinary meatus, and the cleaning time was 30 sec. The method of cleaning is spiral scrubbing from top to bottom. Patients with each disease were divided randomly into the bis in die (BID) group and quaque die (QD) group and started to clean at 24 h and 48 h after surgery. Two q-tips for sampling were used before and after cleaning on the surrounding area of urinary meatus and surface of catheter, one for bacterial culture and drug sensitivity test, and one for further experiments and stored in sterile tube with 5 mL saline under -80°C.

### 2.3. Observation Index

#### 2.3.1. Bacterial Culture

All the samples were used to perform bacterial culture, drug sensitivity test, and 16s rDNA real-time PCR. Some of the samples were performed with 16s rRNA for microbial diversity analysis.

#### 2.3.2. 16s rDNA Real-Time PCR

The DNA copy number of bacteria in each sample was tested by 16s rDNA rt-PCR. The probes are 515F5′-GTGCCAGCMGCCGCGG-3′; 806R,5′—GGACTACHVGGGTWTCTAAT—3′. The experiments were performed by Slan 96P real-time PCR system (Shanghai Hongshi Medical Technology Co., Ltd) and qPCR MIX kit (RR430A, Takara) according to the manufacturer's instructions. The amplification program was set to run at 95°C for 3 min followed by 30 cycles of 30 s of denaturation at 94°C, 20 s of annealing at 60°C, and 20 s of extension at 72°C. pMD19T bacterial 16s was used as the reference standard. The conversion formula of plasmid initial copy number (*copies*/*μl*) = *concentration* (*ng*/*μl*)∗10 − 9∗6.02∗1023∗/*base* *pair*∗324.5∗2.

#### 2.3.3. Microbial Diversity Analysis

Bacterial 16s rRNA gene sequencing of catheter cleaning samples was used for microbial diversity analysis. The probes are 16S V4-V5: 515F-907R, 18S V9: 1380F-1510R, and ITS1: ITS1F- ITS2R. The allocated sequencing region was amplified into specific probe with barcode. All the PCR products were collected by GeneJET Gel Extraction Kit (Thermo Scientific) and quantified by QuantiFluor™-ST (Promega). The sequencing library was set by NEB Next®Ultra™ DNA Library Prep Kit for Illumina (NEB, USA) and sequenced by Illumina MiSeq platform to generate 250 bp/300 bp pair-end reads.

The article "Optimizing the Catheter Care and Maintenance Strategy of Short-Term Catheterization among Hospitalized Patients in Microbiological Approach" was retracted in 2024. Reasons: signs of a paper mill; suspected computer-generated content; unreliable results or conclusions; concerns about the data.

Sequencing read pairs were demultiplexed based on the unique molecular barcodes, and reads were merged. A quality filter was applied to the resulting merged reads and those containing above 0.05% expected errors were discarded. Sequences were stepwise clustered into operational taxonomic units (OTUs) to determine taxonomies. The beta-diversity analysis was performed by the *vegdist* function in R package “vegan” with the method of “bray,” to generate Bray-Curtis distance. The hierarchical clustering was performed using complete linage method to calculate the linkage distances based on the Bray-Curtis distance between samples. Principal Co-ordinates Analysis (PCoA) was performed by the *betadisper* function in R package “vegan.”

### 2.4. Statistical Analysis

Statistical analysis was done using R 3.2.1. Normally distributed data were expressed in mean ± standard deviations (SD) and compared using Student's *t* test; otherwise was indicated as median (Q1~Q3) and compared using the nonparametric Mann-Whitney test. *P* < 0.05 was considered statistically significant.

## 3. Result

A total of 117 male postoperative patients and 54 female postoperative patients were included in this study. The number and age of patients in each operation type is shown below (Table 1). There was no statistical difference between the routine urine examination of patients in all groups before and after cleansing (Table 2).

### 3.1. Detection of the Absolute Number of Bacteria

1. The overall situation of the sample: all patients of various diseases have no significant difference before and after cleansing at 24 hours postoperatively; there is no significant difference between the samples before and after cleansing at 48 hours postoperatively (Table 3). There was no significant difference between the 24-hour and 48-hour postoperatively samples before cleansing (*P* = 0.776 for male; 0.174 for female).
2. The patients' samples after cleansing according to BID are divided into two groups: cleaned before noon (am) and after noon (pm). The results showed that no matter am or pm, there was no significant difference in the total amount of bacteria in the samples before and after cleansing at 24 hours or 48 hours postoperatively (Table 4).
3. Compare within groups according to different disease groups: there is no difference in the samples before and after 24-hour or 48-hour cleansing within each disease group. There was no difference between the samples within the disease group (except for the male calculus group) at 24 hours or 48 hours postoperatively before cleansing. In the male calculus group, the number of bacteria in the samples before cleansing at 24 hours postoperatively was significantly higher than that before cleansing at 48 hours (*P* < 0.001; Table 5).

The article "Optimizing the Catheter Care and Maintenance Strategy of Short-Term Catheterization among Hospitalized Patients in Microbiological Approach" was retracted in 2024. Reasons: signs of a paper mill; suspected computer-generated content; unreliable results or conclusions; concerns about the data.

### 3.2. Bacterial Species Detection

1. The results of bacterial culture were partially consistent with that of 16s rDNA fluorescence quantitative PCR detection distribution (Figures 1-3)
2. Before and after QD cleansing for male at 24 hours postoperatively, the proportion of pathogenic bacteria consistent with the culture results decreased (Figure 1; left 1-2: Staphylococcus), and the proportion of other major types of bacteria did not change significantly
3. For the male group, there was no significant change in the proportion of bacteria and other major types of bacteria consistent with the culture results before and after QD cleansing at 48 hours postoperatively. And there was no significant change in the proportion of major bacterial species before and after BID cleansing at 24 hours no matter cleansing before or after noon (Figures 1, 3(a), and 3(c)).
4. For the female group, the large variation in bacterial species before and after cleansing was mainly due to genital-associated flora rather than urinary tract infections. Therefore, the reference value of the change of bacterial species sampled in the female group remains to be discussed (Figures 2, 3(b), and 3(d)).

## 4. Discussion

According to the guidelines of various countries, it is recommended to clean the inlet and outlet of the urinary catheter 1-2 times a day. Therefore, we cleaned the indwelling catheters at 24 hours and 48 hours postoperatively once a day (QD) and twice a day (BID). The results suggest that although bacterial culture and microbial diversity analysis have a certain consistency in the detection of bacterial species, uncleanness within 48 hours will not cause significant urinary tract bacterial increase, urinary tract infection, and bacteriuria. In addition, there was no significant difference in the samples before and after cleansing for all patients of each disease at 24 hours and 48 hours postoperatively and no significant difference between the samples before cleansing at 24 hours and 48 hours postoperatively, which indicated that no cleansing within 48 hours will not cause significant urinary tract infections. In order to further confirm this conclusion, we conducted a study on the time frequency. Two cleansings (forenoon and afternoon) were performed at 24 or 48 hours postoperatively, and samples were taken before and after the cleansings. There was no significant difference in the total amount of bacteria in the samples before and after cleansing, no matter forenoon and afternoon. In terms of disease types, there was no difference among the groups, which supported this conclusion. However, the calculus group was an exception, the number of bacteria in the sample of patients in this group before the 24 hours cleansing was significantly higher than that before the 48 hours cleansing. The above results are applicable to both male and female patients.

The article "Optimizing the Catheter Care and Maintenance Strategy of Short-Term Catheterization among Hospitalized Patients in Microbiological Approach" was retracted in 2024. Reasons: signs of a paper mill; suspected computer-generated content; unreliable results or conclusions; concerns about the data.

We have found in clinical practice that due to the increase in postoperative urethral secretions and the application of catheter coatings, stains on patients' catheters will form biofilms. Some studies believe that the biofilm formed by bacterial plaque on the catheter is one of the causes of repeated or serious urethral infections [13–15]. If these biofilms are removed in time, it can play a positive role in the prevention of urethral infections caused by catheters. Our results suggest that the biofilm bacterial culture and microbial diversity analysis have a certain consistency in the detection of bacterial species. But results confirm that even if there are secretions in the urethra or biofilms in the catheter within 48 hours postoperatively, the culture results will not show significant infection. Therefore, as such a hidden danger, we are considering whether it is enough to wipe off the plaque on the surface of the catheter.

The evidence basis of the previous clinical nursing cleansing program mainly comes from urine examination and bacterial culture. With the development of molecular biology technology, the evidence-based medical evidence in the past catheter care guidelines has shown certain limitations. We used the microbiological diversity detection technology to obtain accurate biological evidence of catheter samples, so as to further explore and study the cleansing strategy of catheter. We used this technology to test the catheter cleaning fluid and found that whether the catheter was cleaned within 24 to 48 hours postoperatively did not affect the distribution of bacterial species and changes in the number of bacteria on the catheter, nor would it cause CAUTI. The change of bacterial species in the samples of female patients before and after cleansing was limited to the killing of long-term colonized bacteria of the reproductive tract and was not associated with urinary infection. Therefore, cleansing the catheter after 48 hours is a crucial period for short-term indwelling catheter care. In addition, our study also found that after the catheter was not cleaned 72 hours postoperatively, the total copy number of bacteria did not increase significantly. However, the proportion of positive bacteria in bacterial culture increased significantly, and the expansion of the bacterial plaque and changes in color could be observed on the appearance of the catheter, and the number of white blood cells in the urine of patients was also increased. It corroborates the conclusions of previous researchers that the incidence of urinary tract infections has increased significantly since the third day after surgery [16].

The article "Optimizing the Catheter Care and Maintenance Strategy of Short-Term Catheterization among Hospitalized Patients in Microbiological Approach" was retracted in 2024. Reasons: signs of a paper mill; suspected computer-generated content; unreliable results or conclusions; concerns about the data.

## 5. Conclusions

This study conducted an in-depth study on the routine nursing work of indwelling catheterization, suggesting that the cleansing care of indwelling short-term catheterization for patients within 48 hours after urological surgery can be adjusted according to the needs, that is, to reduce the number of mental care or only wipe the secretion or biofilm. It provides a reliable reference basis for promoting the rational allocation and effective use of medical and nursing resources. From the perspective of nursing economy, the research results have greatly saved manpower costs, changed traditional concepts, or nursing strategies, and allowed nurses more time to return to serving patients. But the sample size of this study is not large enough; we will continue to collect samples in the future, expand to more patients, and use more data to verify our conclusions.

## Figures and Tables

**Figure 1:** 16s RNA analysis of different approaches to the cleansing of indwelling catheterization for male. QD: quaquedie; B: bisindie; b: before cleaning; a: after cleaning.

**Figure 2:** 16s RNA analysis of different approaches to the cleansing of indwelling catheterization for female. QD: quaquedie; B: bisindie; b: before cleaning; a: after cleaning.

**Figure 3:** The beta-diversity analysis of the bacterial species between different approaches to the cleansing of indwelling catheterization. The dendrograms based on the Bray-Curtis distances between the samples from male (a) or female (b). The PCoA biplots for the samples from male (c) or female (d).

**Table 1a:** (a) For male

Type of disease	Number	Age (average)
Calculus	24	55.3 ± 14.3
Prostate tumor	23	68.1 ± 6.5
Kidney tumor	19	48.2 ± 12.7
Bladder tumor	22	63.7 ± 14.3
Adrenal tumor	18	54.0 ± 13.3
Prostatic hyperplasia	11	68.5 ± 5.2
Total	117	59.6 ± 13.4

**Table 1b:** (b) For female

Type of disease	Number	Age (average)
Calculus	10	56.5 ± 15.5
Kidney tumor	23	55.4 ± 11.2
Bladder tumor	6	70.2 ± 14.3
Adrenal tumor	15	51.3 ± 11.2
Total	54	58.0 ± 13.05

**Table 2a:** (a) For male

Term	In-hospital	Statistical value	*P* value	Precleaning	Statistical value	*P* value	Postcleaning
Age	59.60 ± 13.40			59.60 ± 13.40			59.60 ± 13.40
Bacterial count (*μ*L)	18.8 (9.1~49.8)	0.225	0.822	20.8 (8.65~40.25)	-0.852	0.396	20.75 (6.73~45.6)
Occult blood (positive %)	56.9	38.231	^∗∗∗^	96.1	0	0.122	100
Tube count (*μ*L)	0.38 (0.128~1.24)	-0.610	0.542	0.43 (0.12~1.26)	-1.692	0.092	0.27 (0.123~0.985)
Red blood cell count (*μ*L)	12.3 (5.2~70.9)	-4.873	^∗∗∗^	262.95 (44.88~972.1)	-0.441	0.658	204.15 (50~834.85)
White blood cell count (*μ*L)	9.3 (3.7~43.2)	-3.121	^∗∗∗^	92.55 (35.43~199.38)	-0.477	0.631	63.6 (36.15~165.5)
Epithelial cell count	3.9 (1.28~7.78)	-0.774	0.44	5.4 (1.9~11.2)	-1.373	0.172	3.7 (2.0~9.43)
Glucose (positive %)	13.89	11.732	^∗∗∗^	38.83	0	1	38.89
Ketosome (positive %)	2.78	14.291	^∗∗∗^	25.24	0.020	0.887	23.33
Leukocyte lipase (positive %)	29.17	50.39	^∗∗∗^	83.50	3.015	1	83.33
Nitrite (positive %)	2.78	1.442	1	1.94	0	0.501	0
pH	6.03 ± 0.57	-5.361	^∗∗∗^	6.50 ± 0.57	0.622	0.536	6.56 ± 0.56
Protein (positive %)	61.11	1.101	0.294	69.90	0.113	0.739	66.67
Urine specific gravity	1.02 ± 0.009	3.368	^∗∗∗^	1.01 ± 0.008	-0.58	0.56	1.01 ± 0.008
Turbidity (turbid %)	86.11	10.137	^∗∗^	64.08	1.050	0.311	71.11
Urobilinogen (negative %)	0	0	0.511	1.94	0.572	1	1.11
Small round epithelial cell (negative %)	0	0	1	0	0.004	0.946	1.10

Statistical values are *t* value for Student's *t* test, *χ*^2^ for chi-square test, and OR value for Fisher test; *P* value: ^∗∗^, <0.01; ^∗∗∗^, <0.001.

The article "Optimizing the Catheter Care and Maintenance Strategy of Short-Term Catheterization among Hospitalized Patients in Microbiological Approach" was retracted in 2024. Reasons: signs of a paper mill; suspected computer-generated content; unreliable results or conclusions; concerns about the data.

Data were shown by mean ± SD or *M*(p25 ~ p75).

**Table 2b:** (b) For female

Term	In-hospital	Statistical value	*P* value	Precleaning	Statistical value	*P* value	Postcleaning
Age	58.00 ± 13.05			58.00 ± 13.05			58.00 ± 13.05
Bacterial count (*μ*L)	75.9 (27.5~542.2)	1.94	0.058	31.6 7.875~70.45)	-1.38	0.17	40.9 (9.4~90.7)
Occult blood (positive %)	56.41	7.54	^∗∗^	84.62	3.86	0.10	95.56
Tube count (*μ*L)	0.38 (0.13~1.20)	-0.19	0.85	0.395 (0.09~1.0125)	-0.76	0.45	0.5 (0.00~0.83)
Red blood cell count (*μ*L)	15 (6.2~38.25)	-2.84	^∗∗^	115.10 (23.05~247.4)	-0.441	0.95	153.75 (27.85~349.2)
White blood cell count (*μ*L)	31.4 (9.3~161.6)	-0.34	0.74	51.65 (16.825~172.975)	0.11	0.91	75.4 (20.8~152.8)
Epithelial cell count	7.0 (3.0~26.0)	2.39	^∗^	4.6 (2.825~7.9)	-0.37	0.71	4.1 (2.3~8.7)
Glucose (positive %)	5.13	0.30	0.18	15.38	0.36	0.55	22.22
Ketosome (positive %)	10.26	0.42	0.52	17.31	0.38	0.54	24.44
Leukocyte lipase (positive %)	58.97	0.001	0.98	61.54	0.0071	0.93	64.44
Nitrite (positive %)	7.69	19.7	^∗∗∗^	0	0	1	0
pH	6.12 ± 0.54	-2.63	^∗^	6.41 ± 0.52	0.63	0.53	6.48 ± 0.49
Protein (positive %)	38.46	0.49	0.48	48.08	0.098	0.75	53.33
Urine specific gravity	1.02 ± 0.007	2.74	^∗∗^	1.01 ± 0.008	-0.29	0.77	1.01 ± 0.008
Turbidity (turbid %)	23.08	0.17	0.68	17.31	0.12	0.73	22.22
Urobilinogen (negative %)	0	0	1	0	0	1	0
Small round epithelial cell (negative %)	0	0	1	0	0	1	0

Statistical values are *t* value for Student's *t* test, *χ*^2^ for chi-square test, and OR value for Fisher test; *P* value: ^∗∗^, <0.01; ^∗∗∗^, <0.001.

The article "Optimizing the Catheter Care and Maintenance Strategy of Short-Term Catheterization among Hospitalized Patients in Microbiological Approach" was retracted in 2024. Reasons: signs of a paper mill; suspected computer-generated content; unreliable results or conclusions; concerns about the data.

Data were shown by mean ± SD or *M*(p25 ~ p75).

**Table 3a:** (a) For male

Postsurgery	b vs. a
24 h	0.840
48 h	0.551

**Table 3b:** (b) For female

Postsurgery	b vs. a
24 h	0.128
48 h	0.284

**Table 4a:** (a) For male

Postsurgery	b vs. a-am	b vs. a-pm
24 h	0.82	0.659
48 h	0.285	0.786

**Table 4b:** (b) For female

Postsurgery	b vs. a-am	b vs. a-pm
24 h	0.533	0.138
48 h	0.652	0.349

**Table 5a:** (a) For male

Type of disease	24 h b vs. a	48 h b vs. a	24 h b vs. 48 h b
Calculus	0.745	0.695	0.001^∗^
Prostate tumor	0.708	0.297	0.309
Kidney tumor	0.786	0.314	0.314
Bladder tumor	0.613	0.505	0.882
Adrenal tumor	0.539	0.935	0.653
Prostatic hyperplasia	0.739	0.902	0.133

**Table 5b:** (b) For Female

Type of disease	24 h b vs. a	48 h b vs. a	24 h b vs. 48 h b
Calculus	0.842	0.549	1
Kidney tumor	0.935	0.4	0.159
Bladder tumor	0.905	NA	NA
Adrenal tumor	0.014^∗^	0.31	0.298

## Data Availability

The original data presented in this study can be inquired from the corresponding authors.

## References

[1] Feneley R. C., Hopley I. B., Wells P. N. (2015). Urinary catheters: history, current status, adverse events and research agenda. *Journal of Medical Engineering & Technology*.

[2] Lam T. B. L., Omar M. I., Fisher E., Gillies K., MacLennan S. (2014). Types of indwelling urethral catheters for short-term catheterisation in hospitalised adults. *Cochrane Database of Systematic Reviews*.

[3] Anderson D. J., Kirkland K. B., Kaye K. S. (2007). Underresourced hospital infection control and prevention programs: penny wise, pound foolish?. *Infection Control and Hospital Epidemiology*.

[4] Hooton T. M., Bradley S. F., Cardenas D. D. (2010). Diagnosis, prevention, and treatment of catheter-associated urinary tract infection in adults: 2009 International Clinical Practice Guidelines from the Infectious Diseases Society of America. *Clinical Infectious Diseases*.

[5] Alessandri F., Mistrangelo E., Lijoi D., Ferrero S., Ragni N. (2006). A prospective, randomized trial comparing immediate versus delayed catheter removal following hysterectomy. *Acta Obstetricia et Gynecologica Scandinavica*.

[6] Griffiths R., Fernandez R., Cochrane Incontinence Group (2007). Strategies for the removal of short-term indwelling urethral catheters in adults. *Cochrane Database of Systematic Reviews*.

[7] Fukuoka K., Furuichi M., Ito K. (2018). Longer duration of urinary catheterization increases catheter-associated urinary tract infection in PICU. *Pediatric Critical Care Medicine*.

The article "Optimizing the Catheter Care and Maintenance Strategy of Short-Term Catheterization among Hospitalized Patients in Microbiological Approach" was retracted in 2024. Reasons: signs of a paper mill; suspected computer-generated content; unreliable results or conclusions; concerns about the data.

[8] SARI (2011). Guidelines for the prevention of catheter-associated urinary tract infection. *Japanese Sociological Review*.

[9] Gould C. V., Umscheid C. A., Agarwal R. K., Kuntz G., Pegues D. A., Healthcare Infection Control Practices Advisory Committee (HICPAC) (2010). Guideline for prevention of catheter-associated urinary tract infections 2009. *Infection Control & Hospital Epidemiology*.

[10] Wong E. S., Hooton T. M. (1981). Guideline for prevention of catheter-associated urinary tract infections. *Infection Control*.

[11] Cheung K., Leung P., Wong Y. C. (2008). Water versus antiseptic periurethral cleansing before catheterization among home care patients: a randomized controlled trial. *American Journal of Infection Control*.

[12] Lo E., Nicolle L. E., Coffin S. E. (2014). Strategies to prevent catheter-associated urinary tract infections in acute care hospitals: 2014 update. *Infection Control and Hospital Epidemiology*.

[13] Bossa L., Kline K., McDougald D., Lee B. B., Rice S. A. (2017). Urinary catheter-associated microbiota change in accordance with treatment and infection status. *PLoS One*.

[14] Xu Y., Moser C., al-Soud W. A. (2012). Culture-dependent and -independent investigations of microbial diversity on urinary catheters. *Journal of Clinical Microbiology*.

[15] Maharjan G., Khadka P., Siddhi Shilpakar G., Chapagain G., Dhungana G. R. (2018). Catheter-associated urinary tract infection and obstinate biofilm producers. *Canadian Journal of Infectious Diseases and Medical Microbiology*.

[16] Nickel J. C., Grant S. K., Costerton J. W. (1985). Catheter-associated bacteriuria. An experimental study. *Urology*.

